# Effect of Early Cognitive Training Combined with Aerobic Exercise on Quality of Life and Cognitive Function Recovery of Patients with Poststroke Cognitive Impairment

**DOI:** 10.1155/2022/9891192

**Published:** 2022-04-12

**Authors:** Haiyu Jiang, Haihong Li, Zheng Wang, Xiaomei Xia, Qinglun Su, Jinya Ma

**Affiliations:** ^1^Department of Rehabilitation Medicine, the First People's Hospital of Lianyungang/the First Affiliated Hospital of Kangda College of Nanjing Medical University, 222061 Lianyungang, Jiangsu, China; ^2^Department of Nursing, the First People's Hospital of Lianyungang/the First Affiliated Hospital of Kangda College of Nanjing Medical University, 222061 Lianyungang, Jiangsu, China

## Abstract

**Objective:**

To explore the effect of early cognitive training combined with aerobic exercise on quality of life (QOL) and cognitive function recovery of patients with poststroke cognitive impairment (PSCI).

**Methods:**

Ninety PSCI patients treated in our hospital from April 2019 to April 2020 were selected as the subjects and were divided into the experimental group (EG) and control group (CG) according to the admission order, with 45 cases each. Patients in CG received conventional health education combined with rehabilitation training, and those in EG accepted early cognitive training combined with aerobic exercise so as to evaluate the clinical effect of different intervention modes on PSCI patients.

**Results:**

Compared with CG after intervention, EG obtained an obviously higher Stroke Specific Quality of Life scale (SS-QOL) score, Montreal Cognitive Assessment (MoCA) score, Barthel Index (MBI) (BI) score and Functional Independence Measure (FIM) score (*P* < 0.001), and obviously shorter time for completing TMT-A and TMT-B (*P* < 0.001).

**Conclusion:**

Performing early cognitive training combined with aerobic exercise for PSCI patients can effectively improve their QOL and promote the recovery of cognitive function. Compared with conventional health education combined with rehabilitation training, this mode presents a higher application value. Further study will be conducive to establishing a better solution for patients.

## 1. Introduction

Epidemiological surveys have shown that stroke is one of the cerebrovascular diseases with high incidence in China, has a high rate of lethality and disability, and ranks first among the lethal/disabling diseases in China [1, 2]. At present, most scholars believe that the disease is related to advanced age, lower education level, stroke condition, and vascular related risk factors such as hypertension, smoking, and atrial fibrillation. Meanwhile, cholinergic system lesions, excitatory neurotransmitter toxicity, oxidative stress, apoptosis, and inflammatory response may contribute to the pathogenesis of the disease. Kapoor Arunima [3] et al. reported that, at present, there are about 6.9 million cases and 1.9 million new cases of stroke in China, and the incidence is increasing at a rate of 8.5%. Betrouni Nacim [4] et al. stated that 1.6 million people died of stroke each year, and stroke accounted for 22.37% of all the causes of death from disease. Meanwhile, it has been reported that more and more younger patients have a stroke in China currently [5]. The prevention and treatment of stroke have become the focus of scholars in the medical community. Impaired cognition is the most significant complication affecting the prognosis and rehabilitation of patients after stroke, the degree of which is more than the pain and inconvenience caused by limb dysfunction to patients. Therefore, more and more foreign and domestic scholars have paid attention to the study of PSCI in recent years [6]. Verstraeten [7] et al. stated that the concern of the World Stroke Day proclamation shifted from disability to PSCI in 2015, and it was clearly suggested that rehabilitation of PSCI should be given high attention. Molad Jeremy [8] et al. reported that the US International Stroke Conference in 2016 proposed to integrate intervention modalities for PSCI, and in the *Guidelines for Adult Stroke Rehabilitation*, the importance of evaluation for PSCI was further emphasized and poststroke cognitive function training was highly recommended.

Stroke is characterized mainly by focal neurological deficits and acute onset, which is a cerebrovascular disease that can cause structural brain abnormalities, with a considerable incidence of PSCI. It has been reported that the global incidence of PSCI ranges from 40% to 70% and that the rate varies depending on the patients' ethnic origin, region, and diagnostic criteria [9]. Baccaro Alessandra [10] et al. indicated that the incidence of PSCI in China was about 80.85%, including 31.87% of poststroke dementia patients and 47.93% of nondementia patients with cognition impairment. The numerous effects of decreased quality of life (QOL), impaired mental health, and even aggravation of disability caused by PSCI lead to great distress for patients. But related reports have pointed out that PSCI is not irreversible and the brain can recover cognitive function through functional reorganization of neural cells, which may be due to certain plasticity of the nervous system [11]. In addition, many published works have confirmed that early cognitive training has a promoting effect on restoring cognitive function in PSCI patients [12]. Moreover, Sanchez-Bezanilla Sonia [13] et al. demonstrated that aerobic exercise also attenuates cognitive impairment and improves QOL in patients with PSCI. But the combination of early cognitive training and aerobic exercise has rarely been reported. Based on this, the combined intervention was adopted for the subjects in this study, in the hope of providing a more clinical evidence-based basis for such patients.

## 2. Materials and Methods

### 2.1. General Data

Ninety PSCI patients treated in our hospital from April 2019 to April 2020 were selected as the subjects and were divided into the experimental group (EG) and the control group (CG) according to their admission order, with 45 cases each. The study met the World Medical Association Declaration of Helsinki (2013) [14].

### 2.2. Enrollment of Subjects

Inclusion criteria. ① The patients met the diagnostic criteria for PSCI in the *Endovascular Management of Cerebrovascular Disease* [15] and were diagnosed after brain CT or MRI examination, with clinical manifestation of reduction of calculation, memory, and executive function; ② the patients had a stable condition and vital signs; ③ the patients had the disease for the first time and a medical history of more than 12 weeks; ④ the patients were 40 to 80 years old; ⑤ the patients did not have aphasia, organic depression, reactive depression, and other diseases and related family history.

Exclusion criteria for the patients. ① The patients had medical history of other diseases that might affect the cognitive function, such as Parkinson's disease, traumatic brain injury, or mental diseases; ② the patients could not go along with the cognitive test and training due to language, movement, or sensation disturbance, etc.; ③ the patients were complicated with severe heart, liver, lung and kidney diseases; ④ the patients were involved in other studies; ⑤ the patients were complicated with severe internal medicine diseases; ⑥ the patients had used psychotropic medication for a long time.

### 2.3. Methods

#### 2.3.1. CG

Conventional health education combined with rehabilitation training was performed on patients in CG. Healthcare workers developed the brochures based on the characteristics of stroke for patients to learn and improve their awareness of stroke pathogenesis, clinical manifestations, treatment modalities, and adverse effects. At the same time, patients were given routine limb training, including muscle passive massage, active movement of joints and affected limbs, balance function training in sitting position, and body transfer, and training on the cognitive levels regarding intelligence, ability of expression, memory, and comprehension was carried out. The intervention was conducted continuously for 6 months.

#### 2.3.2. EG

Early cognitive training. When the patients' vital signs were stable, orientation rehabilitation training was performed to them by the specially engaged rehabilitation therapists, such as frequently reminding patients of the time for going to bed or get up and the movement route of the repeated training. The specific measures were as follows: ① perceptual disturbance rehabilitation training, including sensory integration and visual training, recognizing the shape or color of objects, etc.; ② thought disturbance rehabilitation training, e.g., patients were encouraged to go out, return to the ward, or order food by themselves; ③ memory disturbance rehabilitation training, such as training patients to remember their names, or guiding patients to retell a story; ④ attention deficit rehabilitation training, e.g., showing pictures according to patients' preferences and guiding them to describe the objects in the pictures, once a day and 6 times a week for continuous 6 months; meanwhile, the patients were asked to repeat 1–30 positive and negative numbers and repeat the odd/even numbers respectively; ⑤ orientation training, the therapists asked the patients for time, date and place, and trained the patients to do the addition, subtraction, division and multiplication within the number range of 0 to 50; ⑥ memory training, assisting the patients in remembering the person or objects that they just saw, and, with the help of patients' family members, assisting the patients in recalling the recent events, gaining ability to solve problems, and completing simple tasks independently such as wearing clothes, taking off clothes, and washing the face; ⑦ language training, talking about patients' topic of interest, and raising questions to promote their language ability in solving problems; ⑧ balance function training, the healthcare workers trained the patients in static balance function by using the balance function trainer and assisted the patients in moving on the balance table while keeping balance; meanwhile, during the training period, the healthcare workers should adjust the exercise time and the speed of the training according to the patients' degree of disturbance to 15 min each time, twice a day, and 6 times a week for continuously 6 months.

#### 2.3.3. Aerobic Exercise

In this study, the aerobic exercise was carried out with the ergometric bike for lower limbs (manufacturer: Shanghai Yilian Medical Instrument Development Co., Ltd.; model: E-GLC-02), which was divided into the phases of warm-up, aerobic exercise, and cooling down. ① Warm-up: Prior to training, the patients were assisted in adjusting the seat to a suitable height and guided to maintain the correct position of riding a bike, with both feet placed on the pedals and properly secured with the fixing straps. Before warm-up, the resistance parameters should be adjusted according to the patients' exercise capacity, and the patients were instructed to ride the bike at a relatively slow speed for 6 to 12 min. Before the training started, the patients were taught to repeatedly ride the bike with the unaffected lower limb as the dominating limb to assist the affected limb until they were skillful, so as to provide a good foundation for the aerobic exercise with a certain intensity at a later stage. ② Aerobic exercise: Resistance parameters were adjusted according to the patients' subjective level of fatigue and accommodation to riding the bike. At the same time, 65%–70% of the limit heart rate was set as the training standard throughout the 25 min aerobic exercise, and the patients' vital signs were closely monitored during the training, with careful attention paid to their subjective exercise sensation. ③ Cooling down: When the 25 min aerobic exercise finished, the patients should not stop immediately and should continue to maintain low-intensity bike riding for 6 to 12 min, during which the researcher should gradually reduce the resistance parameter values of the ergometric bike until the end of the exercise. Patients' heart rate and blood pressure during exercise were monitored to timely detect their discomfort symptoms such as nonsubjective chest distress and palpitation. Health education was conducted to the patients and their family members before treatment to inform them on the precautions of aerobic exercise, and the intervention was carried out for 6 months. If patients experience discomfort symptoms during exercise, the training should be promptly discontinued, and further measures should be taken.

### 2.4. Observation Indicators

The Stroke Specific Quality Of Life (SS-QOL) [16] scale was used to evaluate the quality of life (QOL) of patients in the two groups after the intervention, which contained 12 aspects and 49 items, and each item was rated on a scale of 0–5 points, with higher scores indicating better QOL.

The Montreal Cognitive Assessment (MoCA) [17] was used to evaluate the cognitive function of patients in the two groups, which included attention and concentration, executive functions, memory, language, visuoconstructional skills, conceptual thinking, calculations, and orientation. The total score of the scale was 30 points, and scores ≥26 points were regarded as normal cognition. After obtaining the patients' consent and when the patients were conscious, stable, and presented no resistance and suppression, a quiet environment was provided for them to do the test.

The Barthel index (BI) [18] was used to measure the patients' performance in activities of daily living after the intervention, including items such as dressing, grooming, feeding, bathing, toilet use, mobility on level surfaces (45 m on flat ground), walking up and downstairs, and transfer (bed to chair and back). On a scale of 0–100 points, the score was proportional to the patients' ability to perform activities of daily living.

The Trail Making Test (TMT) [19] was a common test for executive function, which included part A and part B and might help identify cognitively impaired patients. In part A, numbers from 1 to 25 were shown on a sheet of paper dispersedly, and the patients should draw lines to connect the numbers in ascending order; in part B, both numbers (1–13) and letters (A - L) were shown on a sheet of paper, and the patients should draw lines to alternatively connect the numbers and letters in ascending order (i.e., 1-A-2-B-3-C, etc.). The shorter the time to finish the tasks, the better the executive function.

The Functional Independence Measure (FIM) [20] was used to evaluate the independence of patients in the two groups after treatment, which contained mobility (self-care, sphincter control, transfers, locomotion, etc.) and cognitive function (communication, social cognition). On a scale of 18–126 points (91 points for mobility and 35 points for cognitive function), higher scores indicated better independence.

### 2.5. Statistical Processing

In this study, the data processing software was SPSS20.0, the picture drawing software was GraphPad Prism 7 (GraphPad Software, San Diego, USA), the items included were enumeration data and measurement data, the methods used were X^2^ test, *t*-test, and normality test, and differences were considered statistically significant at *P* < 0.05.

## 3. Results

### 3.1. Baseline Data

Table 1 showed that no statistical between-group differences in gender, age, BMI value, course of disease, type of stroke, complications, disease site, educational degree, religious faith, family income, and place of residence were observed (*P* > 0.05).

### 3.2. SS-QOL Scores

Figure 1 showed that compared with CG after the intervention, EG obtained a significantly higher SS-QOL score (*P* < 0.001).

Note: The horizontal axis indicated EG and CG, and the vertical axis indicated the SS-QOL score (points). The SS-QOL scores of EG and CG were, respectively, (212.98 ± 8.15) and (170.09 ± 6.40) and indicated a significant between-group difference in SS-QOL scores after intervention (*t* = 27.765, *P* < 0.001).

### 3.3. MoCA Scores

Table 2 showed that compared with CG after the intervention, EG obtained an obviously higher MoCA score (*P* < 0.001).

### 3.4. BI Scores

Figure 2 showed that compared with CG after the intervention, EG obtained an obviously higher BI score (*P* < 0.001).

Note: The horizontal axis indicated EG and CG, and the vertical axis indicated the BI score (points). The BI scores of EG and CG were, respectively, (83.96 ± 1.45) and (65.02 ± 1.34) and indicated a significant between-group difference in BI scores after intervention (*t* = 65.352, *P* < 0.001).

### 3.5. TMT-A and TMT-B Results

Table 3 showed that compared with CG, the time for completing TMT-A and TMT-B was obviously lower in EG (*P* < 0.001).

### 3.6. FIM Scores

Figure 3 showed that compared with CG after the intervention, EG obtained a greatly higher FIM score (*P* < 0.001).

Note: The horizontal axis indicated after intervention, and the vertical axis indicated the FIM score (points); The FIM scores of EG and CG were, respectively, (100.87 ± 7.83) and (68.78 ± 6.43) and indicated a significant between-group difference in FIM scores after intervention (*t* = 21.247, *P* < 0.001).

## 4. Discussion

The cognitive function involves many aspects, such as memory, perception, reasoning, operations, attention, concept formation, problem solving, executive function, language, and information processing speed. When one of them is impaired, the function of the cognitive domain will also decline, such as reduced attention and memory and the inability to discriminate the orientation, and if two or more cognitive domains are impaired, it is considered to have cognitive dysfunction [21]. Cognitive impairment is a common poststroke sequela, and relevant data show that PSCI has a high prevalence in China, with great harm, so early recognition, assessment, and rehabilitation of PSCI are also regarded as a highly important part of stroke medical treatment [22]. At present, clinical routine rehabilitation training is limited to the preaching of stroke pathogenesis and precautions, which has relatively single content, so patients have poor motivation, and long-term training easily causes physical and mental exhaustion of patients, thus reducing their training compliance, leading to the unsatisfactory recovery of their cognitive function and finally affecting QOL. The content of routine education is too specialized and tends to be process-oriented, so patients can only absorb half the information, which results in poor adherence to later treatment. In addition, Rohde Daniela [23] et al. reported that, by absorbing some theories from behavioral science, the American psychologist Rex proposed to perform persuasion and education to patients and remove unjustified beliefs, which achieved effective therapeutic outcomes. Brain functional training, the relearning process of cognitive function, is currently recognized as the best means of cognitive rehabilitation. The plasticity of the central nervous system provides theoretical support for functional training in cognitive rehabilitation, so that the brain can promote the reconstruction of neural networks and functions through the release of various neurotransmitters. Meanwhile, a large number of studies at home and abroad have also confirmed the effectiveness of early cognitive training in cognitive rehabilitation, and its therapeutic effects have been generally recognized by clinicians [24]. And some scholars believe that introducing aerobic exercise on this basis can achieve better clinical outcomes. After 6 months of conventional intervention in this study, the statistical analysis of the SS-QOL scale of the two groups showed that the SS-QOL score was obviously higher in EG than in CG (*P* < 0.001), demonstrating that early cognitive training combined with aerobic exercise played an active role to PSCI and was conducive to promote QOL, which was consistent with the current clinical study results. The reason is that patients are often asked to take an active part in the early cognitive rehabilitation training, which is targeted and recovers their cognitive ability as far as possible and has a promoting effect on improving their QOL. Moreover, aerobic exercise effectively increases the total blood volume, enhances the pulmonary function of patients, improves cardiac function, and greatly promotes the healing process.

Aerobic exercise, featured with long duration, low intensity, and rhythmicity, is the physical exercise conducted when the body is under adequate supply of oxygen, during which the body inhales oxygen equal to the quality demanded to achieve a physiologically balanced state. In recent years, aerobic exercise has gradually attracted more attention due to its role in improving PSCI, but its mechanism to improve cognitive function is still unclear, and some scholars believe that it is mainly through the remodeling of the nervous system. Hung [25] et al. pointed out that aerobic exercise can improve the time course of synaptic transmission of information substances and regulate the decrease in the number of synapses, structurally change the pathological changes, reduce function of synapses, and play a positive role in improving cognitive dysfunction. Neurotransmitters are equally crucial for neural activity, and they are important regulators of cognition and movement in humans. In this study, compared with CG after the intervention, EG obtained an obviously higher MoCA score (*P* < 0.001) and BI score (*P* < 0.001), implying that combining early cognitive training with aerobic exercise can effectively improve the cognitive ability and activities of daily living of PSCI patients. In addition, the study results showed that compared with CG after the intervention, EG had an obviously short time to finish TMT-A and TMT-B (*P* < 0.001) and an obviously higher FIM score (*P* < 0.001), fully proving that the improved cognitive function is conducive to the promotion of independence of PSCI patients, and that the intervention of combining early cognitive training with aerobic exercise is effective.

Shortcomings of the study: First, the selected cases in this study were patients treated in local hospitals, so the source of cases was single, and limited by relevant conditions, the size of samples included was smaller, and the source of samples was restricted and lacked representativeness; second, both early cognitive training and aerobic exercise are nonpharmacological treatment, which is not suitable for applying the blind method to patients, because patients tend to be subjective to the clinical trial results after knowing their corresponding therapeutic measures, thus causing bias in the results; finally, the clinical study still used scales for evaluation, so when patients were answering the questions, there would be certain unavoidable subjectivity and intention, which would also affect the final results of clinical trials to a certain extent. Therefore, the study design should be improved in the future with an expanded sample size, improved grouping, strictly blinded controls, objective evaluation of indicators of cognitive function, etc., to obtain more rigorous and objective data and conclusions.

## Figures and Tables

**Figure 1:** Between-group comparison of SS-QOL scores after intervention ($\bar{\text{x}}$ ± *s*).

**Figure 2:** Between-group comparison of BI scores after intervention ($\bar{\text{x}}$ ± *s*).

**Figure 3:** Between-group comparison of FIM scores after intervention ($\bar{\text{x}}$ ± *s*).

**Table 1:** Between-group comparison of baseline data.

Item	EG (*n* = 45)	CG (*n* = 45)	x^2^/*t*	*P*
Gender			0.047	0.829
Male	28 (62.22%)	27 (60.00%)		
Female	17 (37.78%)	18 (40.00%)		
Age ($\bar{\text{x}}$ ± *s*, years)	58.00 ± 3.13	58.11 ± 2.56	0.182	0.856
BMI (kg/m^2^)	20.58 ± 0.62	20.59 ± 0.58	0.079	0.937
Course of disease ($\bar{\text{x}}$ ± *s*, weeks)	20.71 ± 3.53	20.31 ± 2.65	0.608	0.545
Type of stroke			0.046	0.830
Cerebral hemorrhage	27 (60.00%)	26 (57.78%)		
Cerebral infarction	18 (40.00%)	19 (42.22%)		
Complication			0.045	0.833
Hypertension	21 (46.67%)	22 (48.89%)		
Diabetes mellitus	24 (53.33%)	23 (51.11%)		
Disease site			0.045	0.832
Hemiplegia on the left side	25 (55.56%)	24 (53.33%)		
Hemiplegia on the right side	20 (44.44%)	21 (46.67%)		

Educational degree				

Primary school and junior high school	17 (37.78%)	19 (42.22%)	0.185	0.667
Senior high school and junior college	14 (31.11%)	15 (33.33%)	0.051	0.822
College and above	14 (31.11%)	11 (24.44%)	0.499	0.480
Religious faith			0.053	0.818
Yes	14 (31.11%)	13 (28.89%)		
No	31 (68.89%)	32 (71.11%)		
Family income			0.067	0.796
≥3,000 yuan/(month·person)	35 (77.78%)	36 (80.00%)		
<3,000 yuan/(month·person)	10 (22.22%)	9 (20.00%)		
Place of residence			0.047	0.829
Urban area	27 (60.00%)	28 (62.22%)		
Rural area	18 (40.00%)	17 (37.78%)		

**Table 2:** Between-group comparison of MoCA scores after intervention ($\bar{\text{x}}$ ± *s*).

Group	*n*	MoCA score
EG	45	28.77 ± 1.44
CG	45	21.13 ± 1.52
t		24.477
P		<0.001

**Table 3:** Between-group comparison of TMT-A and TMT-B results ($\bar{\text{x}}$ ± *s*).

Group	n	TMT-A (s)	TMT-B (s)
EG	45	138.04 ± 46.88	172.01 ± 89.01
CG	45	178.95 ± 43.76	259.74 ± 97.13
t		4.279	4.467
P		<0.001	<0.001

## Data Availability

Data to support the findings of this study are available upon reasonable request from the corresponding author.
